# Bioinformatics Analysis for Identifying Differentially Expressed MicroRNAs Derived from Plasma Exosomes Associated with Radiotherapy Resistance in Non-Small-Cell Lung Cancer

**DOI:** 10.1155/2022/9268206

**Published:** 2022-05-31

**Authors:** Lirong Zeng, Guilin Zeng, Zhong Ye

**Affiliations:** ^1^Chengdu Railway Health School, Chengdu, China; ^2^Chengdu Fifth People's Hospital, Chengdu, China

## Abstract

**Objective:**

To explore the differentially expressed microRNAs (DEmiRs) derived from plasma exosomes related to radiotherapy resistance and their corresponding pathways in non-small-cell lung cancer (NSCLC).

**Methods:**

Plasma samples from NSCLC patients were retrieved and analyzed. The patients were divided into 3 groups based on the tumor regression grade criteria, assessed by radiological imaging after radiotherapy. TRG1 referred to tumor shrinkage of ≤30% after radiotherapy, TRG2 as 30% < TRG < 50%, and TRG3 as TRG ≥ 50%. High-throughput sequencing and bioinformatics analysis were used to compare the DEmiRs between the three groups. The miRanda, PITA, and RNAhybrid software were used to identify potential target genes of the DEmiRs. GO function enrichment and KEGG pathway enrichment analyses were performed on the target gene set.

**Results:**

There were 24 DEmiRs (12 were upregulated and 12 downregulated) between the TRG1 and TRG2 groups, 11 between the TRG1 and TRG3 groups (6 upregulated and 5 downregulated), and 35 between the TRG2 and TRG3 groups. The common DEmiRs between the three groups were miR-92a-3p. GO analysis showed that the target genes of the DEmiRs were mainly enriched in unicellular organism processes, cell transformation, cell localization, and their establishment. KEGG enrichment analysis showed that target genes were significantly enriched in the Ras signaling pathway and associated with endocytosis. Among the 135 identified target genes of miR-92a-3p, 4 were involved in the PI3K-Akt signaling pathway (the downstream pathway of the Ras gene) and 3 in the cAMP signaling pathway (the upstream pathway of the Ras gene). Further, 2 other target genes were involved in the Rap1 signaling pathway (the upstream pathway of PI3K-Akt).

**Conclusion:**

By assessing the expression and functional profile of DEmiRs in the plasma exosomes of NSCLC patients after radiotherapy, miR-92a-3p was identified as a promising target affecting radiotherapy outcomes through the Ras signaling pathway.

## 1. Introduction

Lung cancer is one of the most common cancers worldwide and is associated with high mortality [1, 2]. Globally, more than 14.1 million new patients are diagnosed with lung cancer each year, with an estimated 8.2 million deaths every year. Non-small-cell lung cancer (NSCLC) is the primary type of lung cancer, accounting for up to 85% of all lung cancer cases [3]. Current treatments for NSCLC mainly include surgery, chemotherapy, and radiation therapy, of which thoracic radiotherapy is a key therapeutic strategy [4, 5]. However, radical thoracic radiotherapy cannot usually eradicate all tumor cells. Dawe et al. [6] reported that radiotherapy demonstrated unsatisfactory outcomes, with a median survival of 10 months and 5-year survival of only 5% in stage III NSCLC patients. Other studies have shown that the local recurrence rate of NSCLC could be up to 60-70% after conventionally fractionated radiotherapy [7, 8]. Further, patients with radioresistant tumors are at high risk for recurrence and usually have very poor prognoses [9]. The underlying mechanism of radioresistance is very complicated and has been related to the tumor microenvironment, DNA damage repair, radioresistant genes, tumor heterogeneity, and more [10, 11]. Thus, to enhance the radiosensitivity of NSCLC and improve treatment outcomes, it is important to develop novel strategies to understand its underlying pathogenesis and corresponding radiobiology.

With the recognition and development of liquid biopsy, exosomes are increasingly used to investigate novel therapeutic approaches for managing malignant tumors [12]. Exosomes are one of the carriers actively secreted by living cells for intercellular communication, especially noncoding small RNAs due to their stable internal properties and flexible roles in the occurrence and development of tumors [13]. The expression types and amounts of miRNAs are stage-specific and tissue-specific. Tumor cells can express specific miRNAs at specific periods to regulate cell proliferation, migration, apoptosis, and other activities. For example, miR-142-3p has been shown to exert tumor suppressor effects by targeting the RAC1/PAK1 pathway in breast cancer [14]. It was also shown to target HMGB1 and possess potential tumor suppressor effects on non-small-cell lung cancer [15]. However, miRs are also involved in the occurrence and development of tumors and work in the form of clusters. Numerous studies have confirmed the miR-17-92 cluster as a major oncogenic driver or secondary event that enhances the oncogenic process in different cancer types [16, 17]. Lee et al. [18] confirmed that the overexpression of miR-7 could enhance the radiotherapy sensitivity of malignant glioma and breast cancer cells. Guo et al. [19] observed that miR-30a overexpression enhanced the radiotherapy sensitivity of both A549 and H460 lung cancer cells. In regard to treatments, radiotherapy can cause lung cancer cells to overexpress miR-126 to inhibit tumor cell growth [20].

In a study by Zheng et al. [21], the authors studied the mechanisms of radiotherapy and found that the expression of miRNA-21 was closely related to chemoradiotherapy resistance and EGFR-TKI drug resistance in NSCLC. Mao et al. [22] also found that the expression of miR-181a was significantly downregulated in human lung cancer A549 cells. At the same time, the upregulation of miR-181a expression could improve the radiotherapy sensitivity of lung cancer cells by inhibiting the expression of the target gene *NRP1*. However, most of the experiments related to the radiotherapy sensitivity of NSCLC at present were performed using *in vitro* setting and clinical results are limited.

In this study, we used high-throughput sequencing technology to detect miRNAs in the exosomes of peripheral blood of 13 NSCLC patients after radiotherapy. The differentially expressed miRNAs were qualitatively and quantitatively analyzed to identify associated targeted genes that could improve the radiotherapy efficacy of NSCLC patients.

## 2. Materials and Methods

### 2.1. Sample Collection

The clinical data (gender, age, pathological type, TNM stage, concomitant diseases, living habits, imaging data, molecular markers, etc.) of 13 NSCLC patients admitted at the Chengdu Fifth People's Hospital (Chengdu, China) from September 2017 to March 2019 were collected. Before treatment, the patients underwent biopsy and were diagnosed with NSCLC by the pathology department. All patients included in this study did not receive radiotherapy in previous stages, and their initial treatments were nonsurgical. At admission, their median cubital venous blood was collected before radiotherapy. Their tumor volume, before and after radiotherapy, were assessed using computed tomography (CT) imaging, and the change in tumor volume was graded using the tumor regression grade (TRG) criteria [23]. Briefly, tumors that shrank by ≤30% after radiotherapy were classified into the TRG1 group, and those that shrank between 30% and 50% and ≥50% were classified into the TRG2 and TRG3 groups, respectively. Informed consent was obtained from the patients or their families prior to treatment. The study protocol was approved by the Ethics Committee of Chengdu Fifth People's Hospital (Approval number: SCCHEC-02-2017-030).

### 2.2. Plasma Exosome Enrichment and Plasma Exosome RNA (Exo-RNA) Extraction

The plasma exosomes of each group of patients were gradually extracted according to the instructions of ExoQuick kit (System Biosciences, Mountain View, CA) [24]. Total exosomal RNA extraction was performed on isolated exosomes using the SeraMir™ Exosome RNA Amplification Kit (Cat. # RA810A/TC-1, System Biosciences, USA) following the manufacturer's protocol. After isolation, RNA purity and quantitative analysis was performed on an Agilent Bioanalyzer 2100 system (Agilent Company, USA).

### 2.3. Exo-RNA cDNA Library Construction

After the extracted samples were qualified, the Illumina's NEB Next Multiplex Small RNA Library (NEB, USA) was used to prepare the centralized small RNA libraries. Using the unique structures at the 3′ and 5′ ends of the small RNA, total RNA was used as the starting sample, and both ends of the small RNA were directly added with adapters with cDNA synthesized by reverse transcription. Subsequently, after qPCR amplification, DNA fragments of length 140-160 bp were separated by polyacrylamide gel (PAGE) electrophoresis with the cDNA library recovered by cutting the gel. The Qubit 2.0 was then used for preliminary quantification. The effective concentration of the library was accurately quantified by the qPCR method to ensure library quality. The library quality was evaluated using the Agilent Bioanalyzer 2100 system (Agilent Company, USA) and a DNA high-sensitivity chips.

### 2.4. High-Throughput Sequencing of Plasma Exo-RNA

After the library detection was qualified, the materials of different libraries were combined following the requirements of effective concentration and target off-machine data volume. Then, the index-coded samples were clustered on the cBot cluster generation system using the TruSeq SR Cluster Kit v3 cBot-HS (Illumina, USA). After clustering, the library preparations were sequenced using the Illumina HiSeq 2500 sequencer and 50 bp platform (Illumina, USA). The obtained sequencing data was examined for error rate distribution. After data quality control of the off-machine data, data with a length of 18-30 nt were selected from the clean reads and were compared with the human reference database miRBase 20.0 database (http://www.mirbase.org/) to find matching sRNAs. Non-miRNA databases such as RepeatMasker and Rfam were compared to eliminate known non-miRNAs (repetitive sequences, rRNA, tRNA, snRNA, and snoRNA) and mRNA degradation fragments. The obtained data was then classified and annotated for normalized expression analysis.

### 2.5. miRNA Target Gene Prediction

TargetScan (http://www.targetscan.org/vert_72/), PITA (https://genie.weizmann.ac.il/pubs/mir07/mir07_data.html), and RNAhybrid (https://bibiserv.cebitec. uni-bielefeld.de/rnahybrid/) were used to predict target genes of differentially expressed miRNAs. A Venn plot was constructed for the three groups of results to analyze the correspondence between miRNAs and target genes.

### 2.6. Gene Ontology (GO) Analysis and Kyoto Encyclopedia of Genes and Genomes (KEGG) Analysis

GO (http://www.geneontology.org/) is a widely used bioinformatics tool for enrichment analysis of gene sets, including biological process, cellular component, and molecular function [25]. KEGG (http://www.genome.jp/kegg/) is a database used to investigate the enrichment pathways of selected genes to understand the functions of genes [26]. Using the DAVID database (http://david.abcc.ncifcrf.gov/) [27], GO enrichment and KEGG pathway enrichment analyses were performed separately for the sets of target genes of each group of differentially expressed miRNAs. Functional analysis was also performed on the coexpressed differentially expressed genes to investigate their related cellular components, molecular functions, biological processes, and signaling pathways. *P* values < 0.05 and Count > 2 were used as the enrichment thresholds.

### 2.7. Statistical Analysis

The target genes of the miRNAs were counted using the RNA-seq analysis software. The measure transcripts per million (TPM) was used to estimate miRNA expression levels based on the following criteria: normalized expression = mapped read count/total reads∗1,000,000.

For samples with biological replicates, differential expression was analyzed using the “limma” R software package [28] for each group of both conditions. The adjusted *P* < 0.05 and |log Fold Change (FC)| > 0.8 were regarded as differentially expressed miRNAs. *P* < 0.05 after the correction was considered statistically significant.

## 3. Results

### 3.1. General Information

In all, 13 patients were eligible for this study. Of them, the tumor of 7 patients was classified as adenocarcinoma and 6 as squamous cell carcinoma (Table 1). Their plasma samples were pooled for sequencing and were analyzed. Based on the CT findings after radiotherapy, 4 patients were classified into the TRG1 group, 6 into the TRG2 group, and 3 into the TRG3 group.

### 3.2. Analysis of Differentially Expressed miRNAs Associated with Tumor Regression Volume

The differentially expressed miRNAs were compared between the TRG1 and TRG2 groups, TRG1 and TRG3 groups, and TRG2 and TRG3 groups before radiotherapy. The results showed that there were 24 common differentially expressed miRNAs between the TRG1 and TRG2 groups, 11 between the TRG1 and TRG3 groups, and 35 between the TRG2 and TRG3 groups (Figure 1(a)). Among them, between the TRG1 and TRG2 groups, 12 differentially expressed miRNAs were significantly upregulated and 12 were significantly downregulated in the TRG1 group (Figure 1(b) and Table 2). By comparing the preradiotherapy plasma samples of the TRG1 and TRG3 groups, we observed that 6 differentially expressed miRNAs were upregulated and 5 were downregulated genes in the TRG1 group (Figure 1(c) and Table 3). Further analyses showed that the common differentially expressed miRNA in the three groups was miR-92a-3p (Tables 2 and 3), and it was significantly higher expressed in the TRG1 group.

### 3.3. Targeted Gene Results of Differential miRNAs

The TargetScan, PITA, and RNAhybrid software were used to identify target genes of the differentially expressed miRNAs, and overlapped genes were used for further analysis. The results identified 135 potential target genes (i.e., *ENSG00000079432* and *ENSG00000112852*) for the highly expressed miR-92a-3p in the TRG1 group. After conversion, *CIC*, *PCDHB2*, and other targeted genes were obtained. In the TRG2 group, we identified 50 potential target genes for the highly expressed miR-1307-5p, of which *CDH23* and *LRFN1* were obtained after conversion. Further, 87 potential target genes (i.e., *ENSG00000110104* and *ENSG00000102837*) were identified for miR-151b, 170 genes (i.e., *ENSG00000131203* and *ENSG00000102057*) for the highly expressed miR-205-5p, 139 genes (i.e., *ENSG00000053254* and *ENSG00000167964*) for the highly expressed miR-210-3p, and 291 genes (i.e., *ENSG00000035664* and *ENSG00000100412*) for the highly expressed miR-664b-5p. In the TRG3 group, we identified 288 potential target genes (i.e., *ENSG00000101082* and *ENSG00000103023*) for the lowly expressed miR-27a-5p, 3 potential target genes (*ENSG00000172209*, *ENSG00000172209* and *ENSG00000203778*) for the highly expressed miR-215-5p, 44 potential target genes (i.e., *ENSG00000072195* and *ENSG00000115956*) for the highly expressed miR-24-1-5p, and 4 potential target genes (i.e., *ENSG00000135974* and *ENSG00000144455*) for the highly expressed miR-548a-3p. The gene targeted by the highly expressed miR-548p was ENST00000422289. In addition, we also identified 19 potential target genes (i.e., *ENSG00000079616* and *ENSG00000175556*) for miR-96-5p and 74 potential target genes (i.e., *ENSG00000157368* and *ENSG00000101441*) for the highly expressed miR-96-5p.

### 3.4. Gene Enrichment Analysis

The identified potential target genes of the differentially expressed miRNAs were subjected to GO and KEGG enrichment analyses. GO analysis showed that the biological processes of differentially expressed miRNAs targeting genes between the TRG1 and TRG2 groups were mainly enriched in unicellular organism processes, cell transformation, cell localization, and establishment. The cellular components were localized into intracellular components, organelles, organelles with membrane structure, and more. The molecular functions were enriched in protein binding, bonding, and molecular functions (Figure 2(a)). Before radiotherapy treatment, the biological processes of differentially expressed miRNA-targeted genes between the TRG1 and TRG3 groups were mainly enriched in cellular localization and establishment, metabolic process, small molecule metabolism, etc. The cellular components were localized into the intracellular components, cytoplasm, organelles with membrane structure, etc. Further, the molecular functions were enriched in protein binding, bonding, enzymatic reactions, etc. (Figure 2(b)).

Specific analyses revealed that differentially expressed miRNA target genes between the TRG1 and TRG2 groups were enriched in cellular process, cell, molecular functions, etc., while those between the TRG1 and TRG3 groups were enriched in metabolic processes, intracellular, binding, etc. The enrichment intersection of the three groups was for protein binding.

KEGG enrichment analyses showed that differentially expressed miRNAs targeting genes between the TRG1 and TRG2 groups were significantly enriched in the Ras signaling pathway and endocytosis (Figure 2(c)). The KEGG pathways of 135 genes targeted by miR-92a-3p were analyzed, of which 4 target genes were found to be involved in the PI3K-Akt signaling pathway, 3 target genes in the cAMP signaling pathway (the upstream pathway of Ras gene), and 2 target genes in the natural killer cell-mediated cytotoxicity (natural killer cell cytotoxic activity pathway). Further, 2 target genes were observed to be involved in the Rap1 signaling pathway (upstream pathway of PI3K/Akt), 2 target genes in autophagy, and 2 target genes in cell cycle, and 1 target gene was directly involved in the Ras signaling pathway.

## 4. Discussion

The exosome-derived miRNAs in circulating blood are stable in structure, have flexible expression, and have significant tissue and time specificities [29]. The expression of miRNAs is closely related to the sensitivity of lung cancer radiotherapy [30]. miR-92a-3p is an essential member of the miR-17-92 cluster [31]. The miR-17-92 cluster is reported to have tumor suppressor or tumor-promoting roles in different types of tumors. In NSCLC, the expression of miR-92a-3p was found to be relatively higher in more advanced clinical stages [32]. It has been previously reported that miR-92a-3p could promote esophageal squamous cell carcinoma proliferation, migration, and invasion by targeting PTEN [33]. The exosome miR92a-3p was shown to promote the epithelial-to-intercellular transition and metastasis of low-metastatic hepatocellular carcinoma cells by regulating the PTEN/Akt pathway [34]. In colon cancer, it was able to directly downregulate DIckkopf-3 (Dkk-3) with the help of extracellular vesicles (EVs) to promote angiogenesis, upregulate the endothelial cell cycle, and promote mitosis in endothelial cells to induce angiogenesis [35]. In lung cancer, miR-92a-3p could promote the proliferation and migration of lung cancer cells, A549, through NF2 [36]. Roudkenar et al. [37] used clinically relevant radiation-resistant (CRR) cell experiments to demonstrate that miR-17-92 cluster and HIF-1*α* synergistically promoted the radioresistance of CRR cells. Thus, high expression of the miR-17-92 cluster has been demonstrated to be associated with reduced radiotherapy sensitivity in CRR cells. In this study, the only common differentially expressed miRNA between the three TRG groups was miR-92a-3p. In comparison, the expression of miR-92a-3p in the TRG1 group was significantly higher than that of the other two groups. Therefore, since patients in the TRG1 groups had the poorest response to radiotherapy, we hypothesized that miR-92a-3p could have been one of the important factors affecting the efficacy of radiotherapy in NSCLC patients and could thus be regarded as a promising biological marker for radioresistance in NSCLC.

The Ras gene family mainly contains 3 types of genes: *H-ras*, *K-ras*, and *N-ras*. Mutations of the *ras* gene in human tumors often occur at codons 12, 13, 59, or 61, and different tumors have predominant differences in the activation of the three *ras* genes [38, 39]. Lung cancer is mainly dominated by *K-ras* mutations, which enhance the self-amplification characteristics of NSCLC cancer cells through nuclear-transcribed gene activity and affect the clinical outcomes of patients [40, 41]. The Ras protein expressed by the activated Ras gene affects the controlled regulation of GTP and GDP. The activated Ras protein continuously activates PLC to generate second messengers, resulting in uncontrollable cell proliferation, malignant transformation, and reduction of apoptosis [42]. The upstream pathways of Ras are complicated and can be activated by receptors such as EGFR and PDGFR, which require the binding of various proteins such as Grb2, Sos, and C3G [43]. Ras activation can maintain cell survival through the PI3K/Akt pathway.

In this study, KEGG enrichment analysis of differentially expressed miRNA target genes in the three groups indicated that the differentially expressed miRNA target genes were significantly enriched in the Ras signaling pathway. GO analysis of the molecular functions of TRG was enriched in protein binding and bonding, and the gene function nodes were enriched in protein binding. The above results suggest that the difference between TRG1 and the TRG2 and 3 groups could be genetically distinct from protein binding and bonding in the Ras pathway. Screening of plasma exosome-derived miRNAs in the three TRG groups showed that only miR-92a-3p was the common differentially expressed between them. KEGG analysis of its target genes revealed that multiple genes of miR-92a-3p were directly or indirectly involved in the PI3K/Akt pathway, and multiple genes were closely related to the upstream and downstream of the Ras signaling pathway. Therefore, we hypothesized that the highly expressed miR-92a-3p in the TRG1 group reduced the efficacy of NSCLC radiotherapy by targeting the Ras pathway.

## 5. Conclusion

In conclusion, high-throughput sequencing technology was used to screen differentially expressed miRNAs in the exosomes of circulating blood of NSCLC patients who had different responses to radiotherapy. miR-92a-3p was identified as a tumor-promoting factor for NSCLC. It weakened the radiotherapy efficacy of NSCLC patients by acting on the Ras pathway through multiple target genes and the PI3K-Akt downstream pathway. Thus, miR-92a-3p could be considered a promising predictor of radiotherapy efficacy in NSCLC.

## Figures and Tables

**Figure 1:** Screening of differentially expressed genes. (a) Venn plot of common differentially expressed genes. (b) Volcano plot of the differentially expressed miRNAs of the TRG1 and TRG2 groups. (c) Volcano plot of the differentially expressed miRNAs of the TRG1 and TRG3 groups.

**Figure 2:** Functional enrichment analysis of differentially expressed miRNA target genes. (a) GO analysis of the TRG1 and TRG2 groups. (b) GO analysis of the TRG1 and TRG3 groups. (c) KEGG enrichment analysis.

**Table 1:** Sample grouping.

Clinical features		Tumor regression volume (TRG) grouping		
		TRG ≤ 30%	30% < TRG < 50%	TRG ≥ 50%
Pathological type	Adenocarcinoma	3	3	1
	Squamous cell carcinoma	1	3	2
Mean age		64	61.8	56
Clinical phase	I phase	1	0	0
	III phase	1	3	1
	IV phase	2	3	2

**Table 2:** Differentially expressed miRNAs between the TRG1 group and TRG2 group before treatment.

sRNA	Read count TRG1	Read count TRG2	log_2_FoldChange	Regulation	*P* value
miR-92a-3p	6351.541	2447.145	1.1854	Up	0.004421
miR-200b-3p	142.8446	51.26118	1.2086	Up	0.008744
miR-574-3p	112.3857	58.57962	0.88466	Up	0.009713
miR-656-3p	13.45293	2.184043	1.5165	Up	0.01043
miR-25-3p	7286.578	3634.27	0.90318	Up	0.012151
miR-373-3p	5.129287	0	1.3052	Up	0.013628
miR-6837-5p	2.056854	0	1.2357	Up	0.020334
miR-429	14.28389	5.191157	1.1444	Up	0.022535
miR-7110-3p	3.449376	0.266368	1.3202	Up	0.024318
miR-615-3p	7.118875	0.727064	1.1777	Up	0.041967
miR-302a-3p	2.738243	0	0.99719	Up	0.0434
miR-1180-3p	109.8191	33.21246	1.1425	Up	0.044635
miR-210-3p	26.22435	76.97575	-1.2791	Down	0.002504
miR-363-3p	1517.85	2544.614	-0.71516	Down	0.002537
miR-483-5p	4.034501	19.28374	-1.5696	Down	0.004539
miR-664b-5p	1.848978	9.490666	-1.517	Down	0.005124
miR-151b	13.4447	34.67708	-1.0293	Down	0.008886
miR-205-5p	2.781506	18.98065	-1.4921	Down	0.010896
miR-23a-5p	17.02933	49.21838	-1.1897	Down	0.015982
miR-24-2-5p	236.1747	466.18	-0.87114	Down	0.019296
miR-339-3p	192.0291	449.7415	-1.0086	Down	0.026063
miR-766-5p	24.82181	46.56813	-0.77471	Down	0.035131
miR-326	68.1303	150.2219	-0.93312	Down	0.038886
miR-1307-5p	44.65798	108.9963	-0.98242	Down	0.044102

**Table 3:** Differentially expressed miRNAs between the TRG1 group and TRG3 group before treatment.

sRNA	Read count TRG1	Read count TRG3	log_2_FoldChange	Regulation	*P* value
miR-34c-5p	15.8276	1.120492	1.5064	Up	0.022304
miR-449c-5p	8.265883	0.263553	1.4729	Up	0.024415
miR-27a-5p	78.25364	14.98098	1.4166	Up	0.025728
miR-11400	239.5607	39.61981	1.4392	Up	0.026697
miR-3928-3p	15.64795	2.471396	1.3884	Up	0.029003
miR-92a-3p	5278.554	2007.793	1.089	Up	0.044564
miR-96-5p	13.79805	61.22625	-1.6069	Down	0.007731
miR-24-1-5p	10.60856	45.27693	-1.52	Down	0.009676
miR-215-5p	13.24125	56.14516	-1.5055	Down	0.012773
miR-548a-3p	7.245361	54.73202	-1.6032	Down	0.014713
miR-548p	7.550065	56.21549	-1.5811	Down	0.016186

## Data Availability

The data used to support the findings of this study are available from the corresponding author upon request.
